# miR-206 Inhibits Laryngeal Carcinoma Cell Multiplication, Migration, and Invasion

**DOI:** 10.1155/2021/5614861

**Published:** 2021-11-26

**Authors:** Yiling Liu, YunTao Song, Xiaojuan Chen, Junfang Fan, Wei Zheng, Chen Cao

**Affiliations:** ^1^Department of Otorhinolaryngology, The Second Affiliated Hospital of Zhengzhou University, Zhengzhou, Henan 45000, China; ^2^Department of Nursing, The Second Affiliated Hospital of Zhengzhou University, Zhengzhou, Henan 45000, China; ^3^Department of Surgery, The Second Affiliated Hospital of Zhengzhou University, Zhengzhou, Henan 45000, China; ^4^Dean's Office, The Second Affiliated Hospital of Zhengzhou University, Zhengzhou, Henan 45000, China; ^5^Department of Intervention, The Second Affiliated Hospital of Zhengzhou University, Zhengzhou, Henan 45000, China

## Abstract

Laryngeal carcinoma (LC) is one of the common human cancer types. MicroRNAs (miRNAs) were reported to be the essential regulators in cancer diagnosis, treatment, and prognosis. It was reported that miR-206 expression was reduced in various neoplastic diseases. However, the role and functional mechanism of miR-206 in LC progression remain unclear. In this research, miR-206 was found to be associated with tumor-node-metastasis (TNM) staging. In addition, the area under the curve (AUC) of miR-206 was 0.902 for diagnosis of LC and 0.854 for differential diagnosis of stage I-II and stage III-IV patients. Low expression of miR-206 was associated with poor prognosis of LC patients. miR-206 expression was an independent factor affecting the prognosis of LC patients, as revealed by the Cox regression analysis. *In vitro* experiments demonstrated that miR-206 overexpression reduced cell multiplication, invasion, and migration and increased cell apoptosis in LC cells. Moreover, SOX9 was a target of miR-206, and miR-206 negatively regulated SOX9 expression. Collectively, miR-206 might be a promising biomarker with diagnostic and prognostic value for LC, and the miR-206/SOX9 axis might be a candidate target for LC therapy.

## 1. Introduction

Laryngeal carcinoma (LC) is a malignancy with the highest incidence among head and neck cancers and accounts for 1%–5% of human cancer types [1]. According to the Global Cancer Statistics 2018, the prevalence of LC was 3.6 and 0.5 per 100,000 in men and women, respectively. Moreover, the mortality rate of LC occupied 1% of total cancer mortality [2]. Most LC patients were diagnosed at the advanced stages with high invasiveness due to the atypical early clinical presentations [3]. Although surgery and radiotherapy could improve the life expectancy of LC patients, approximately 30% of them suffered from recurrence or metastasis. Tumor invasion and metastasis were the main causes for the poor survival rate of LC patients [4]. It was known that drinking and smoking were the most important risk factors of LC [5]. In addition, some researchers found that the family history of cancer was also a risk factor of LC, suggesting that genetic factors also affected LC progression [6]. Thus, it was of value to explore the potential target for the therapy of LC.

As the endogenous noncoding single-stranded small RNA molecules, microRNAs (miRNAs) widely exist in the organisms [7]. miRNAs are the essential regulators in the biological processes and act as oncogenes or antioncogenes in various tumor processes, including cell apoptosis, metastasis, invasion, multiplication, differentiation, and angiogenesis [8]. miRNAs were proved to play crucial roles in various malignancies [9, 10]. Interestingly, miR-206 was verified to be downregulated in various tumors [11]. For example, miR-206 negatively regulated the expression of KIF2A and was related to the worse prognosis in ovarian carcinoma patients [12]. Moreover, miR-206 could inhibit hepatocyte growth factor-induced cell epithelial-mesenchymal transition and angiogenesis in non-small-cell lung cancer via the c-Met/PI3k/Akt/mTOR pathway [13]. A recent research reported that decreased miR-206 was observed in oral cancer and miR-206 might be an effective diagnosis biomarker at an early stage of oral cancer [14]. In hepatocellular carcinoma, miR-206 was demonstrated to exert regulatory effect on the function of cancer stem cells [15]. More importantly, it was reported that miR-206 was involved in the progression of laryngeal squamous cell carcinoma [16]. A previous study showed that miR-206 was dramatically reduced in the tissues of laryngeal squamous cell carcinoma and decrease of miR-206 accelerated the progression of laryngeal squamous cell carcinoma through regulating the expression of VEGF [17]. Moreover, miR-206 overexpression depressed cell proliferation in Hep-2 cells by targeting cyclin D2, and upregulation of miR-206 could inhibit tumor growth in the mice model of laryngeal squamous cell carcinoma [18]. However, the role and underlying mechanism of miR-206 in LC progression are still poorly understood.

In this research, we determined the level of miR-206 in serum and cells of LC patients and found that miR-206 was significantly downregulated in LC. Moreover, our results demonstrated that miR-206 suppressed cell growth, metastasis, and elevated cell apoptosis in LC cells. Besides, we analyzed the association between miR-206 level and the clinicopathological features of LC patients. The data showed that miR-206 level was correlated with tumor-node-metastasis (TNM) staging, suggesting that miR-206 might be a potential diagnostic indicator for LC. Furthermore, we observed that LC patients with a low level of miR-206 exhibited a worse survival rate. Overall, these findings displayed that miR-206 played a suppressive role in LC development, providing a possible diagnosis and prognosis biomarker for LC.

## 2. Materials and Methods

### 2.1. Clinical Samples

This research followed the principles in the Declaration of Helsinki and was ratified by the internal Ethics Committee of the Second Affiliated Hospital of Zhengzhou University. All participants provided the written informed consent. 68 pairs of LC and para-carcinoma tissues were collected from 68 LC patients who underwent surgical resection at the Second Affiliated Hospital of Zhengzhou University and stored at −80°C. These patients were diagnosed with LC by histology or pathology [19]. According to the TNM Classification of Malignant Tumors, 29 LC patients were classified as stage I-II and 39 LC patients as stage III-IV [20]. According to the WHO classification of tumors, 33 LC patients were classified as high/moderate differentiation and 35 LC patients as low differentiation [21]. The LC patients did not receive radiotherapy or chemotherapy. 68 healthy volunteers were also recruited. Plasma samples were collected from 68 LC patients and 68 healthy volunteers. Overall survival (OS) started from diagnosis date to death date or the end of the follow-up. Participants were enrolled from March 2013 to January 2016. The clinicopathological features of these LC patients are presented in Table 1.

### 2.2. Cell Culture and Transfection

The normal bronchial epithelial 16HBE cell lines and LC cell lines (TR-LCC-1 and SNU899 cells) provided by ATCC (Manassas, VA, USA) were cultivated in RPMI medium 1640 (Thermo Fisher Scientific, Shanghai, CHN) containing 10% fetal bovine serum (FBS) and 100 U/mL penicillin/streptomycin at 37°C with 5% CO_2_. For cell transfection, TR-LCC-1 and SNU899 cells (1 × 10^6^ cells/mL) were seeded into the 12-well plates. The miR-206 mimics (miR-206 mim) and the negative control (NC-mim), and miR-206 inhibitor (miR-inh) and the negative control (NC-inh) were synthesized by BGI Genomics (Shenzhen, China) and transfected into TR-LCC-1 and SNU899 cells using Lipofectamine 2000 (Invitrogen, Carlsbad, CA, USA).

### 2.3. Real-Time Quantitative Polymerase Chain Reaction (RT-qPCR)

Total RNA was extracted using TRIzol kits (Invitrogen), and the purity of total RNA was determined using a NanoDrop 1000 spectrophotometer (Thermo Fisher Scientific, Wilmington, DE, USA). Then, the PrimeScript miRNA cDNA reagent (Takara, JPN) was utilized for inverse transcription of RNA into cDNA. RT-qPCR was performed on a 7500HT rapid real-time PCR system (Thermo Fisher Scientific, Shanghai, CHN) using the SYBR Premix Ex Taq II kit (Takara, JPN) following the manufacturer's protocol. The relative expression was calculated using the 2−^ΔΔCT^ method, with U6 or GAPDH as the standardized control. Primer sequences: miR-206 sense: 5′-CCACACACTTCCTTACATTCCATAA-3′, antisense: 5′-CCTCTTACCTCAGTTACAATTTATA-3′; SOX9 sense: 5′-AGGTGCTCAAAGGCTACGACTG-3′, antisense: 5′-CCTAATGTTCATGGTCGGCGC-3′; U6 sense: 5′-CTCGCTTCGGCAGCACA-3′, antisense: 5′-AACGCTTCACGAATTTGCGT-3′; GAPDH sense: 5′-GATCATCAGCAATGCCTCCT-3′, antisense: 5′-TGAGTCCTTCCACGATACCA-3′.

### 2.4. Western Blot

The proteins were extracted using RIPA, and the protein concentration was detected by the Bradford method. The proteins were then separated using SDS-PAGE (10%) and transfected to a PVDF membrane. Then, the membrane was incubated with 5% skim milk for 2 h, followed by incubation with the primary antibodies against SOX9 (1 : 1,000) and GAPDH (1 : 2,000) overnight at 4°C and the horseradish peroxidase-labeled specific secondary antibody (1 : 5,000) at room temperature for 2 h. Finally, the protein bands were visualized using the ECL reagent and the gray value of the protein bands was analyzed using Image J. The fold change was calculated by GAPDH normalization. The antibodies were provided by Abcam, Cambridge, UK.

### 2.5. Cell Multiplication Assay

Cell multiplication was measured using the CCK-8 kit (Fuyuan Biotech, Shanghai, CHN) following the manufacturer's protocol. TR-LCC-1 and SNU899 cells were seeded on the 96-well plates and treated with 10 *μ*L of CCK-8 solution. The optical density (OD) was analyzed at 450 nm using the Varioskan LUX multifunctional microplate reader (Thermo Fisher Scientific, Waltham, MA, USA).

### 2.6. Transwell Migration and Invasion Assays

Cell migration and invasion abilities were determined using Transwell inserts (Thermo Fisher Scientific, Waltham, MA, USA), and Matrigel (BD Biosciences, San Jose, CA, USA) precoated on a Transwell chamber was utilized for cell invasion capacity measurement. 1 × 10^5^ TR-LCC-1 and SNU899 cells in serum-free RPMI medium 1640 were added in the upper chamber, and 600 *μ*L RPMI medium 1640 containing 10% FBS was placed in the lower chamber. Then, the migrated or invaded TR-LCC-1 and SNU899 cells were dyed with crystal violet solution for 5 min and counted using an inverted microscope. The average number of cells was calculated in five randomly selected fields under the microscope.

### 2.7. Dual-Luciferase Reporter Assay (DLRA)

Target genes of miR-206 were predicted using TargetScan (http://www.targetscan.org/), a target gene prediction database, and the binding sites between miR-206 and SOX9 3′UTR were found. The wild-type (WT) or mutant (MUT) segments of SOX9 harboring the complementary sites of miR-206 were cloned into the pGL3 vector (Promega, Madison, WI, USA) to form WT-SOX9 and MUT-SOX9 luciferase reporter vectors. Then, WT-SOX9, MUT-SOX9, NC-mim, and miR-206 mim were cotransfected into the cells using Lipofectamine 2000 (Invitrogen). Luciferase activity was measured after 48 h transfection.

### 2.8. Statistical Methods

The data were shown as the mean ± SD, and differences were analyzed the *t*-test and Chi-square test. The Pearson correlation coefficient was obtained for correlation analyses. The efficacy analysis of miR-206 in LC diagnosis was performed by the receiver operating characteristic curve (ROC). The Kaplan–Meier method was utilized for survival statistics, and Cox regression was employed to analyze the prognostic factors of LC. Difference with *P* < 0.05 was deemed significant. The data were analyzed by SPSS 17.0 and visualized by GraphPad 6.0 software.

## 3. Results

### 3.1. miR-206 Was Downregulated in LC Patients

RT-qPCR revealed that miR-206 was notably reduced in LC tissues compared with the para-carcinoma normal tissues (Figure 1(a)). Serum miR-206 was lower in LC tissues than that in the para-carcinoma normal tissues (Figure 1(b)). We found that miR-206 expression in tissues was positively related to the level of miR-206 in serum by the Pearson correlation coefficient (*r* = 0.822, *P* < 0.001, Figure 1(c)). Moreover, miR-206 was significantly decreased in LC cells compared with the 16HEB cells (Figure 1(d)). These results suggested that miR-206 might be a tumor inhibitor in LC progression.

### 3.2. Low Expression of miR-206 Was Related to the Poor Prognosis of LC Patients

The connection between the clinicopathological features and serum miR-206 levels in LC patients is presented in Table 1. Clinical data showed that miR-206 expression was closely associated with TNM staging, but not related to gender, age, differentiation degree, tumor diameter, tumor location, and history of smoking (Table 1). Serum miR-206 was lower in LC patients with TNM stage III-IV than in patients with stage I-II (Figure 2(a)). ROC curve analysis further evaluated the diagnostic ability of miR-206 in LC, and miR-206 could distinguish TNM staging. Serum miR-206 was able to distinguish LC patients from healthy controls, with the diagnostic AUC of 0.902 (95% CI (confidence interval) = 0.852–0.951; Figure 2(b)). In addition, the AUC of serum miR-206 in differentiating stage I-II patients from stage III-IV was 0.854 (95% CI = 0.767–0.941; Figure 2(c)). Subsequently, survival analysis was performed to further evaluate the ability of serum miR-206 in prognosis. Kaplan–Meier analysis identified a greatly reduced 5-year survival rate in LC patients with low serum miR-206 expression compared with the LC patients with high miR-206 expression (Figure 2(d)). Serum miR-206 might be a valuable biomarker for the diagnosis and prognosis of LC.

### 3.3. miR-206 Acted as a Prognostic Indicator in LC Patients

The clinical characteristics in univariate analysis were gender, age, TNM staging, differentiation degree, tumor diameter, tumor location, and smoking history. Univariate Cox regression analysis indicated that TNM staging and serum miR-206 were strongly bound up with overall survival in LC patients (Tables 2 and 3). In addition, TNM staging and serum miR-206 expression were independent factors that affected the prognosis of LC patients. The relative risk (RR) of serum miR-206 level to overall survival was 3.831, and the 95% confidence interval was 1.065–13.779.

### 3.4. miR-206 Inhibited LC Cell Multiplication, Invasion, and Migration and Promoted LC Cell Apoptosis

To study the potential function of miR-206 in LC, CCK-8 and Transwell assays were used to analyze the impact of miR-206 on LC cell multiplication, migration, and invasion. Our data indicated that miR-206 was remarkably upregulated in TR-LCC-1 cells after miR-206 mim transfection, while miR-206 inh transfection significantly decreased miR-206 expression in SNU899 cells (Figure 3(a)). CCK-8 assay revealed that miR-206 overexpression could inhibit the multiplication of TR-LCC-1 cells, while miR-206 knockdown could promote the multiplication of SNU899 cells (Figure 3(b)). Meanwhile, miR-206 overexpression dramatically reduced cell apoptosis in TR-LCC-1 cells, while miR-206 knockdown enhanced cell apoptosis in SNU899 cells (Figure 3(c)). Transwell assays demonstrated that miR-206 overexpression repressed cell migration and invasion in TR-LCC-1 cells, while miR-206 knockdown enhanced cell migration and invasion in SNU899 cells (Figures 3(d) and 3(e)). All these findings revealed the antitumor role of miR-206 in the progression of LC.

### 3.5. SOX9 Was a Direct Target of miR-206

Next, we further explored the underlying mechanism of miR-206 in LC. TargetScan predicted the binding sites between SOX9 and miR-206 (Figure 4(a)). Then, we verified the potential connection between miR-206 and SOX9 by DLRA. The luciferase activity was evidently reduced by miR-206 mim in the SOX9 3′UTR WT group, but not in the SOX9 3′UTR Mut group (Figure 4(b)). In addition, SOX9 protein expression was suppressed by miR-206 overexpression and SOX9 protein expression was enhanced by miR-206 knockdown (Figure 4(c)). RT-qPCR analysis revealed that SOX9 was notably increased in LC (Figure 4(d)). Moreover, an inverse connection between miR-206 expression and SOX9 expression was identified by the Pearson correlation coefficient (Figure 4(e)). The above data indicated that miR-206 could regulate SOX9 expression in LC cells.

## 4. Discussion

Previous literature studies reported that miRNAs functioned as activators or inhibitors in tumor multiplication and metastasis [22]. miR-206 was confirmed to play the inhibition role in some tumors [23]. miR-206 was proved to be downregulated in colorectal cancer and targeted Bcl-2 to mediate chemical resistance, multiplication, and apoptosis of colorectal cancer cells [24]. Besides, miR-206 expression was decreased in prostate cancer tissues and cells, which could suppress cell multiplication and migration and block the cell cycle by targeting CXCL11 in prostate cancer [25]. In addition, lowly expressed miR-34a and miR-206 were closely related to the short overall survival of cervical carcinoma patients [26]. Similarly, we found that miR-206 was reduced in LC tissues, cells, and serum, indicating that miR-206 played a vital role in LC. Moreover, we investigated the connection between serum miR-206 and clinical characteristics. Our data indicated that patients with low expression of miR-206 predicted a late TNM staging of LC. These results suggested that miR-206 might be a tumor suppressor in LC progression.

Recently, miRNAs were extensively studied as the promising biomarkers for cancer detection [27]. Increasing evidence revealed that specific miRNAs might act as the diagnostic or prognostic biomarkers in cancers [28]. The research of Zhang et al. demonstrated that reduced serum miR-133b and miR-206 levels in osteosarcoma patients were associated with the positive metastasis and recurrence of patients, which might cause the poor overall survival [29]. Our research showed that serum miR-206 had a good diagnostic efficacy for LC and a diagnostic value for advanced TNM staging. Thus, we speculated that serum miR-206 might be related to the prognosis of LC patients. Moreover, our data demonstrated that low miR-206 expression that predicted the short overall survival of LC patients was an independent prognostic biomarker. These findings suggested that miR-206 might be a diagnosis and prognosis biomarker in LC.

MiRNAs could regulate various biological processes, thereby participating in the progression of tumors [30, 31]. In this study, we found that miR-206 overexpression attenuated cell multiplication, migration, and invasion and facilitated cell apoptosis, indicating that miR-206 might play an anticancer role in LC. These results were in line with the research of Yu et al., who reported that miR-206 was reduced in LC cells and could repress human laryngeal squamous cell carcinoma cell growth via modulating cyclin D2 [32]. Another research by Zhang et al. indicated that miR-206 could inhibit cell multiplication and invasion through targeting SOX9 in non-small-cell lung cancer [33]. SOX9, a proved carcinogen, was highly expressed in various cancers [34]. The results in this study displayed that SOX9 was highly expressed in LC. Moreover, TargetScan predicted that miR-206 contained the potential binding sites with SOX9. DLRA demonstrated that SOX9 was a direct target of miR-206. Overall, miR-206 might directly target SOX9 to regulate the biological behaviors in LC. Nevertheless, there were still some shortcomings in our research. For example, the effects SOX9 on LC cell behaviors were not obtained. Furthermore, animal experiments were needed to clarify the mechanism of the miR-206/SOX9 axis *in vivo*. In the future research, we will focus on the detailed mechanism of the miR-206/SOX9 axis in LC.

In conclusion, our results revealed that miR-206 was lessened in LC, which might be a diagnosis and prognosis biomarker for LC. In addition, the miR-206/SOX9 axis was involved in the progression of LC, providing a potential target for LC therapy.

## Figures and Tables

**Figure 1:** miR-206 was downregulated in tissues, serum, and cells of LC patients. (a) Measurement of miR-206 expression in tumor tissues and the adjacent normal tissues of LC patients by RT-qPCR. (b) Detection of miR-206 expression in serum of LC patients and healthy controls by RT-qPCR. (c) Correlation of miR-206 expression in serum and tissues of LC patients. (d) Determination of miR-206 expression in 16HBE, TR-LCC-1, and SNU899 cells by RT-qPCR. ^*∗*^*P* < 0.05.

**Figure 2:** Low expression of miR-206 was related to the poor prognosis of LC patients. (a) Serum miR-206 expression in LC patients with different TNM stages by RT-qPCR. (b) The ROC curve of serum miR-206 in diagnosis of LC patients. (c) The ROC curve of serum miR-206 in differentiating TNM staging. (d) Visualization of the overall survival of LC patients with high or low miR-206 expression. ^*∗*^*P* < 0.05.

**Figure 3:** miR-206 inhibited the multiplication, invasion, and migration and promoted cell apoptosis in LC cells. (a) RT-qPCR analysis of miR-206 expression after transfection of miR-206 mim or miR-206 inh. (b) Measurement of cell multiplication by CCK-8 assay. (c) Detection of cell apoptosis by flow cytometry. (d, e) Determination of cell migration and invasion by Transwell assay. ^*∗*^*P* < 0.05.

**Figure 4:** SOX9 was a direct target of miR-206. (a) Potential binding sites of miR-206 and SOX9. (b) Dual-luciferase reporter assay. (c) Western blot detection of SOX9 protein expression after transfection of miR-206 mim or miR-206 inh. (d) RT-qPCR analysis of SOX9 expression in LC. (e) The expression of miR-206 was negatively correlated with SOX9 in LC. ^*∗*^*P* < 0.05.

**Table 1:** Correlation of serum miR-206 expression with clinical characteristics of patients.

Clinicopathological parameters	*n*	miR-206			*P*
		High expression (*n* = 34)	Low expression (*n* = 34)	*t*/*F*	
Gender				1.308	0.253
Male	52	24 (70.59)	28 (82.35)		
Female	16	10 (29.41)	16 (17.65)		
Age (years)				2.147	0.143
<60	38	22 (64.71)	16 (47.06)		
≥60	30	12 (35.29)	18 (52.94)		
TNM staging				7.275	0.007
I-II	29	20 (58.82)	9 (26.47)		
III-IV	39	14 (41.18)	25 (73.53)		
Differentiation degree				1.472	0.225
High/moderate differentiation	33	19 (55.88)	14 (41.18)		
Low differentiation	35	15 (44.12)	20 (58.82)		
Tumor diameter (cm)				0.541	0.462
>3	39	21 (61.76)	18 (52.94)		
≤3	29	13 (38.24)	16 (47.06)		
Tumor location				0.569	0.451
Supraglottic type	25	14 (41.18)	11 (32.35)		
Glottic type	43	20 (58.82)	23 (67.65)		
History of smoking				0.971	0.324
No	28	16 (47.06)	12 (35.29)		
Yes	40	18 (52.94)	22 (64.71)		

**Table 2:** Assignment.

Variables	Assignment
Gender	Male = 1, female = 2
Age (years)	<60 = 1, ≥60 = 2
TNM staging	I-II = 1, III-IV = 2
Differentiation degree	High/moderate differentiation = 1, low differentiation = 2
Tumor diameter (cm)	<3 = 1, ≤3 = 2
Tumor location	Supraglottic type = 1, glottic type = 2
History of smoking	No = 1, yes = 2
miR-206	High miR-206 expression = 1, low miR-206 expression = 2

**Table 3:** Univariate and multivariate Cox analyses of variables for the overall survival of patients with laryngeal carcinoma.

Parameters	Relative risk (95% CI) of overall survival	*P*
Univariate		
Gender	1.351 (0.483–3.777)	0.566
Age (years)	1.19 (0.47–3.016)	0.713
TNM staging	7.679 (1.78–33.133)	0.006
Differentiation degree	1.401 (0.556–3.532)	0.475
Tumor diameter (cm)	0.395 (0.151–1.036)	0.059
Tumor location	0.733 (0.298–1.803)	0.499
History of smoking	1.861 (0.672–5.155)	0.232
miR-206	6.329 (1.848–21.672)	0.003
Multivariate		
TNM staging	4.587 (1.004–20.944)	0.049
miR-206	3.831 (1.065–13.779)	0.04

## Data Availability

The labeled datasets used to support the findings of this study are available from the corresponding author upon request.
